The article "Ovarian-type epithelial tumours of the testis: immunohistochemical and molecular analysis of two serous borderline tumours of the testis" was published in 2015. Journal: Diagn Pathol.

# Ovarian-type epithelial tumours of the testis: immunohistochemical and molecular analysis of two serous borderline tumours of the testis

**DOI:** 10.1186/s13000-015-0342-9

**Published:** 2015-07-22

**Authors:** Tobias Bürger, Hans-Ulrich Schildhaus, Reinhard Inniger, Joachim Hansen, Peter Mayer, Stefan Schweyer, Heinz Joachim Radzun, Philipp Ströbel, Felix Bremmer

**Affiliations:** Institute of Pathology, University Medical Center, Univeristy of Göttingen, Göttingen, Germany; Gemeinschaftspraxis Pathologie, Starnberg, Germany; Praxisgemeinschaft Pathologie, Düsseldorf/Gummersbach, Germany; Department of Urology, Catholic Clinics Oberberg, Engelskirchen, Germany

**Keywords:** Serous borderline tumour, Testis, Immunohistochemistry, KRAS, BRAF-V600E, CGH

## Abstract

Tumours of ovarian-epithelial type of the testis, including serous borderline tumours, represent very rare entities. They are identical to the surface epithelial tumours of the ovary and have been reported in patients from 14 to 68 years of age. We describe two cases of a 46- and a 39-year old man with incidental findings of intratesticular masses of the left respectively right testis. Under the assumption of a malignant testicular tumour the patients were subjected to inguinal orchiectomy. Histologically, the tumours were identical to their ovarian counterparts: They showed a cystic configuration with a fibrous wall and irregular papillary structures lined by partially multistratified columnar cells and areas of hobnail cells. Furthermore, there was mild cytological atypia with a proliferative activity of below 5 % as proved by Ki67 staining; mitoses could not be detected. Immunohistochemically, the tumour cells displayed expression of pan-cytokeratin AE3, progesterone receptor, Wilms’ tumour protein (WT1), and PAX8 (Paired box gene 8). Estrogen receptor was expressed in one case. Octamer-binding transcription factor-4 (OCT4), calretinin, thrombomodulin, and D2-40 were not expressed. Mutation testing of *BRAF* revealed a *BRAF V600E* mutation in one case, while testing for *KRAS* mutations proved to be negative in both. The *BRAF* mutated tumour showed strong cytosolic and membranous positivity for B-Raf also on immunohistochemical analysis. Comparative genomic hybridization of one case could not reveal any chromosomal aberrations.

## Background

Tumours of ovarian epithelial types of the testis represent rare entities, which histologically resemble their ovarian counterparts [1–3]. They have been reported in patients from 14 to 68 years of age and usually present as a scrotal enlargement [4]. In this case report we describe two cases of serous borderline tumours of the testis in a 46- and a 39-year old patient. We will illustrate the clinicopathologic characteristics and the results of *BRAF* and *KRAS* mutation analysis. In addition we performed comparative genomic hybridization (CGH) of one case.

## Case presentations

### Case 1

A 46-year-old man presented in the urological clinic with painless heaviness of the left testis. Urological examinations showed an intratesticular mass of approximately 2 cm in diameter. On ultrasonography this mass proved to be cystic and solid. The tumour markers were not increased. Under the assumption of a malignant testicular tumour an inguinal orchiectomy was performed. The macroscopic inspection of the surgical specimen, which consisted of testis and testicular appendages, presented a total weight of 23 g and a size of 5 × 4.5 × 3 cm. The cut surface of the testis showed an intraparenchymal, circumscribed formation of cystic appearance with a diameter of 1.4 cm and whitish color.

### Case 2

A 39-year-old man showed an intratesticular mass of approximately 1.5 cm in diameter on urological examinations. The tumour markers were not increased. Under the assumption of a malignant testicular tumour an inguinal orchiectomy was performed. The surgical specimen, which consisted of testis and testicular appendages, presented a total weight of 30 g and a size of 6 × 4 × 3.5 cm. The cut surface of the testis showed an intraparenchymal, circumscribed tumour of cystic appearance with a diameter of 2 cm.

### Histology

Microscopic examination of testicular sections confirmed the cystic nature of the lesions, which were lined by a fibrous capsule (Fig. 1a) and contained residues of clear fluid. Intraluminal, irregular papillary structures lined by partially multistratified columnar cells and areas of hobnail cells could be seen. The tumour cells exhibited eosinophilic cytoplasm, the nuclei showed predominantly dense chromatin with prominent nucleoli (Fig. 1b-f). Furthermore, there was mild cytological atypia but no mitoses (Fig. 1g + h). Psammoma bodies could not be detected. Proliferative activity revealed by Ki67 staining was below 5 % in both cases (Fig. 2a). Immunohistochemical examination of the tumour cells displayed expression of pan-cytokeratin AE3 (Fig. 2b), estrogen- and progesterone receptor (Fig. 2c-d), Wilms’ tumor protein (WT1), and PAX8 (Paired box gene 8). The *BRAF* mutated tumour showed strong cytosolic and membranous positivity for B-Raf. Octamer-binding transcription factor-4 (OCT4), calretinin, thrombomodulin and D2-40 were not expressed. The histological findings supported the diagnosis of a serous borderline tumour. The tumour-free testicular tissue displayed regular tubules with intact spermatogenesis and normal interstitial tissue. A Fallopian tubal metaplasia in the paratesticular epithelial structures or ovarian stroma could not be detected. An overview of the immunohistochemical analysis is listed in Table 1.

**Fig. 1:** Serous borderline tumour of the testis: Ultrasound examination shows an unilocular cyst with intracystic papillae (**a**). Histologically, the tumour shows papillary structures encased by a fibrous wall with cystic areas filled with clear fluid (**b**; x20). The tumour cells present with mild cytologic atypia and eosinophilic cytoplasm, the nuclei show a predominantly dense chromatin with prominent nucleoli (**c**; x40 and **d**; x100; **e**, x200; **f**, x200; **g**, x400; **h**, x600)

**Fig. 2:** Serous borderline tumour of the testis: The Ki67 staining exhibits low proliferative activity (**a**; ×100); Lining Epithelial tumour cells express pan-Cytokeratin AE3 (**b**; x200), estrogen receptor (**c**; x400), progesterone receptor (**d**; x400), and PAX8 (**e**; x100). The tumour with *BRAF* mutation shows immunohistochemical B-Raf positivity (**f**, x400). Mutatation analysis revealed a *BRAF V600E* (c.1799 T > A) mutation in one case (**g**)

**Table 1:** Immunohistochemical analyses

	CK	ER	PR	PX8	WT1	TM	CAL	D2	OCT	Ki	Br
Case 1	+	60 %	40 %	+	+	-	-	-	-	<5 %	+
Case 2	+	-	5 %	+	+	-	-	-	-	<5 %	-

*CK* cytokeratin, *ER* estrogenreceptor, *PR* progesteronreceptor, *PX8* PAX8, *WT1* Wilms’ tumor protein, *TM* thrombomodulin, *CAL* calretinin, *D2* podoplanin, *OCT* OCT4, *Ki* Ki67, *Br* serine/threonine-protein kinase B-Raf

### *BRAF* and *KRAS* mutation analysis

DNA was isolated from the formalin-fixed and paraffin embeded tumour tissue with InnuPure-Kit and the InnuPure C16 according to the manufacturer’s protocol (Analytik Jena, Jena, Germany). Mutation analyses of both samples were carried out with pyro-sequencing using the Pyromark Q24 (QIAGEN, Hilden, Germany). For KRAS analysis the therascreen KRAS Pyro Kit CE 24 T and therascreen RAS extension Pyro Kit (both QIAGEN) were used. For BRAF analysis the therascreen BRAF Pyro Kit (QUIAGEN) was used. Sequencing was performed according to manufacturer’s protocol. Mutation analysis of *BRAF* revealed a *BRAF V600E* (c.1799 T > A) mutation in one case. *BRAF* codon 464–469 revealed a wild type. Testing for *KRAS* mutations in exon 2–4 proved to be of wild type in both tumours (Fig. 2e). The clinicopathologic data and cytogenetic findings are listed in Table 2.

**Table 2:** Clinicopathologic data and cytogenetic findings

	Age	Chromosomal alterations (CGH)	*BRAF V600E*	*KRAS*
Case 1	46	none	c.1799 T > A	WT
Case 2	39	none	WT	WT

*CGH* comparative genomic hybridization, *WT* wild type

### Comparative genomic hybridization (CGH)

CGH was performed as described previously [5]. Comparative genomic hybridization, which was carried out in only one of the tumours due to a lack of tissue, could not detect any chromosomal aberrations.

## Discussion

The similarities of male and female germ cell tumours are well known and have been described numerous times in the medical literature. Conversely, there is little information about the much rarer tumours of ovarian epithelial type of the testis and paratesticular tissue. The most commonly observed among these are serous tumours with the majority being of borderline malignancy [6–8, 2, 1, 9]. Invasive carcinoma has to be excluded by the presence of accentuated cellular atypia, necrosis, and stromal invasion. Therefore, extensive sampling of all cases of borderline tumour should be carried out.

It is still a matter of discussion, whether ovarian-type epithelial tumours of the testis originate from the remnants of Müllerian ducts in paratesticular connective tissue, epididymis, and spermatic cord or from Müllerian metaplasia of the mesothelium of the tunica vaginalis testis. The latter theory is supported by the frequent finding of metaplastic serous Müllerian epithelium in these tumours [10]. Likewise, a Müllerian metaplasia of intratesticular mesothelial inclusions, possibly triggered by injury during embryogenesis, is also imaginable [11].

One of the key questions in the diagnosis of ovarian-type epithelial tumours is their distinction from clinically aggressive neoplasms such as mesothelioma of the tunica vaginalis testis and carcinoma of the rete testis. Besides histological features of mesothelioma such as a low cellularity and the absence of psammoma bodies, immunohistochemical mesothelial markers such as D2-40, thrombomodulin, and calretinin can prove to be helpful for this purpose. Serous tumours, for the most part, show an opposite immunohistochemical pattern for those antigens and express ovarian epithelial tumour markers such as epithelial membrane antigen (EMA), CA-125 (cancer antigen 125), cytokeratin 7, CD15 (Leu-1), and Ber-EP4. The immunohistochemical expression of PAX8 (Paired box gene 8) in ovarian-type epithelial tumours is also a very valuable tool for the distinction as it is only rarely traceable in malignant mesothelioma [12]. Wilms’ tumor protein (WT1) is regularly expressed not only in malignant mesotheliomas but also in ovarian serous carcinomas and thus is not suitable to distinguish these tumour entities. Rare differential diagnoses comprise local spread of adenocarcinoma of the rete testis and adenocarcinoma of the epididymis. Typical histological features of serous borderline tumours that were also present in our cases are their cystic nature and papillary budding, which led to the exclusion of adenocarcinoma of the rete testis and epididymis. Furthermore, no foci of stromal invasion could be detected.

Several authors have shown chromosomal aberrations, of which the most frequent were gains of chromosomes 2q, 6q, 5, 8q and 12 and losses of 1p, 17p, 19 and 22q [13–18] in sets of borderline tumours of the ovary using comparative genomic hybridization (CGH). However, only half of the analyzed cases showed any chromosomal changes at all. CGH of one of the testicular borderline tumours was not able to detect any aberrations, which is in concordance with the studies on ovarian specimen and the overall low-grade nature of the lesion.

The *BRAF*-protooncogene is a downstream mediator of *KRAS* and the substitution of valine (V) to glutamic acid (E) at the position 600 of the amino acid sequence causes its most common activating mutation (T1799A). Several authors have shown the mutation of *BRAF V600E* and its detection by mutation analysis and immunohistochemistry in both serous borderline tumours and low-grade invasive carcinoma of the ovary [19, 20]. Mutations in either *BRAF* or *KRAS* can frequently be seen in low grade serous adenocarcinoma and borderline tumours of the ovary and seem to be mutually exclusive [21]. However, high-grade carcinomas usually feature a different genetic profile with mutations of TP53 and NRAS [22]. To our knowledge only one very recent study has shown a mutation of *BRAF V600E* in a serous borderline tumour of the testis [23]. This, together with our findings, supports a common pathogenesis in serous borderline tumours of both female and male.

## Conclusions

Ovarian-type epithelial tumours of the testis are extremely rare and not well studied tumour entities. The detection of a *BRAF*-mutation, which is common in ovarian serous borderline tumours, points to a common pathogenesis of these entities in both genders. Because the differential diagnosis of these tumours includes malignant entities such as mesothelioma and carcinoma of the rete testis, the correct diagnosis, possibly aided by genetic markers, is important for the optimal management.

## Consent

Written informed consent was obtained by patient for publication of this report and any accompanying images. A copy of the written consent is available for review by the Editor-in-Chief of this journal.
